# Gene expression profiling analysis of hepatocellular carcinoma

**DOI:** 10.1186/2047-783X-18-44

**Published:** 2013-11-14

**Authors:** Deyong Kong, Heming Chen, Weiqun Chen, Shuiyi Liu, Hui Wang, Tangwei Wu, Hongda Lu, Qingzhi Kong, Xiaodong Huang, Zhongxin Lu

**Affiliations:** 1 Department of Medical Laboratory, Central Hospital of Wuhan, Wuhan 430014, China; 2 Department of Cardiovascular and Thoracic Surgery, Second Xiangya Hospital, Central South University, Changsha 410078, China; 3 Department of Central Laboratory, Central Hospital of Wuhan, Wuhan 430014, China; 4 Cancer Research Institute of Wuhan, Wuhan 430014, China; 5 Department of Oncology, Central Hospital of Wuhan, Wuhan 430014, China

**Keywords:** Bioinformatics method, Gene expression profiling, Hepatocellular carcinoma

## Abstract

**Background:**

Primary hepatocellular carcinoma (HCC) is one of the most common malignancies in the world. However, the molecular pathogenesis of HCC is not well-understood, and the prognosis for patients with HCC remains very poor.

**Methods:**

To disclose detailed genetic mechanisms in hepatocellular carcinoma (HCC) with a view toward development of novel therapeutic targets, we analyzed expression profiles HCCs and their corresponding noncancerous tissues by using bioinformatics method.

**Results:**

In this paper, we report the identification of genes whose expression has been altered and the changed bio-pathways during hepatocarcinogenesis. Hepatoma cells infect intracellular and intercellular signal transduction through Focal adhesion and cause abnormal expression of important intracellular signaling pathway. In addition, it is worth mentioning that some small molecules still restored to the state similar to normal cells, such as bambuterol and lovastatin. This member gene set would serve as a pool of lead gene targets for the identification and development of novel diagnostic and therapeutic biomarkers to greatly improve the clinical management of HCC patients with different risks of recurrence after curative partial hepatectomy.

**Conclusions:**

The study has great significance for gene therapy and pharmacotherapy and provides a new treatment entry point and a potential new clinical drug for HCC patients.

## Background

Primary hepatocellular carcinoma (HCC) is one of the most common malignancies in the world [1]. The causes of HCC are better understood than those of other cancers in humans. The major risk factors for HCC are chronic hepatitis and exposure to various exogenous carcinogens, including aflatoxin B1 [2]. However, the molecular pathogenesis of HCC is not well-understood, and the prognosis for patients with HCC remains very poor. Like other cancers, HCC demonstrates diverse biological phenotypes, such as proliferation rate, ability to invade vessels and so forth. So, gene expression profiling analysis of HCC provides a clue to clarifying the detailed mechanisms of hepatocarcinogenesis and discovering target molecules for the development of novel therapeutic drugs.

Classic *in vivo* carcinogenesis experiments reveal a higher susceptibility to HCC in male rodents [3-5]. These findings suggest that biologic features of the tumor may differ significantly between the sexes, but the reasons remain unclear. In a recent study, investigators hypothesized that estrogen inhibits the induction of interleukin 6 produced by Kupffer cells [6]. That the serum level of interleukin 6 is elevated in several cancers has been confirmed [7,8].

In this paper, we report the identification of genes whose expression has been altered and the changes in biopathways during hepatocarcinogenesis. The changes in mitogen-activated protein kinase (MAPK) signaling pathways, T-cell receptor signaling pathway, transforming growth factor β (TGF-β) signaling pathway and neurotrophin signaling pathway changed the apoptosis pathway and hematopoietic cell lineage pathways, so that the liver cells showed a unique pathology. In addition, it is worth mentioning that some small molecules were restored to a state similar to normal cells after treatment with agents such as bambuterol and lovastatin. This has great significance for gene therapy and pharmacotherapy and provides a new treatment entry point and a potential new clinical drug for HCC patients.

## Methods

### Gene expression profiles of hepatoma cells and normal cells

In order to explore the differentially expressed genes and possible pathogenesis mechanisms in hepatoma cells compared to normal cells, we collected hepatoma cells and normal cells from different individuals, then we performed DNA microarrays and obtained the genetic profiles. The appropriate expression profiling was researched and obtained from the public functional genomics data repositories Gene Expression Omnibus (GEO) (http://www.ncbi.nlm.nih.gov/geo/) and the European Molecular Biology Laboratory–European Bioinformatics Institute (EMBL-EBI) ArrayExpress. All gene microarrays of hepatoma cells consisted of 32 gene microarrays of hepatoma cells from the GPL96 platform in ArrayExpress and 10 gene microarrays of normal cells from ArrayExpress. GEO data are based on the Affymetrix GPL571 platform data (Affymetrix Human Genome U133A 2.0 Array). We downloaded the original Affymetrix CEL files and the platform probe annotation information file for the next step in bioinformatics analysis.

### Extraction of differentially expressed genes

Microarray data were analyzed using the R software (v.2.13.0) platform [9]. First, we normalized the different chips by robust multichip averaging [10] and then compared them with the difference using the linear regression model package limma [11] to get the differentially expressed genes between the different treatments.

### Gene Ontology analysis of differentially -expressed genes

In order to find the changes and function enrichment of differentially expressed genes at the cellular level, we used the Gene Ontology (GO) database [12] to classify the gene function and location information. We performed GO clustering analysis using the clusterProfiler software package [13,14], then deduced the affinity of these differentially expressed genes to the cells by clustering the cells within their molecular functions and biological processes.

### Biopathways data analysis

In order to understand the metabolic changes that occur in hepatoma cells at the cellular level, we obtained the metabolic and nonmetabolic pathways from the Kyoto Encyclopedia of Genes and Genomes (KEGG) PATHWAY database, which is authoritative, and made use of the Database for Annotation, Visualization and Integrated Discovery website (DAVID; http://david.abcc.ncifcrf.gov/) to analyze the differentially expressed genes using the method of KEGG PATHWAY cluster [9,14] for the changed pathways involved in the hepatoma cells.

### Little molecular expression profiling data analysis

The Connectivity Map (cmap) database contains the expression data of the genomewide transcription of human cells in the activity of small-molecule intervention, including the 6100 group of small-molecule interference experiments (small interfering group and normal control group) and the expression profile of 7056 [15]. We analyzed gene expression differences between normal cells and hepatoma cells and compared the differentially expressed genes caused by these small interfering expression genes with the hope of identifying similar gene expression profiles of normal cells and hepatoma cells or, vice versa, a small interfering group. The differentially expressed genes of normal cells and hepatoma cells were divided into two categories: upregulation and downregulation. We obtained an enrichment value which stands for similarity through Gene Set Enrichment Analysis compared with the differentially expressed genes in the cmap database dealing with small molecules, whose value was between −1 and 1. The closer they were to 1, the more the small molecules were able to simulate the state of normal cells. The closer they were to −1, the more the small molecules were able to simulate the state of the hepatoma cells.

## Results

### Identifying the genes expressed differently in various pathological states

We used the classic *t*-test to examine the expression profiles of hepatoma cells and normal cells and obtained the differentially expressed genes of hepatoma cells. We calculated *P*-values for all genes by performing a *t*-test. The *P*-values were calculated and then adjusted using the Benjamini–Hochberg (BH) method. Selecting a BH *P* value <0.05 as the significance threshold, the expression of 9,775 gene probes were changed, relating to 4,470 genes.

### Gene Ontology clustering of differentially expressed genes

Cellular components, molecular functions and biological processes were individually assessed by analyzing GO clustering on differentially expressed genes, and in each kind of function we obtained the most significant 10 terms, as shown in Tables 1, 2 and 3, respectively.

**Table 1:** Gene Ontology clustering of cellular components

**Cellular component**	**False discovery rate**
[GO:0000267] Cell fraction	4.69E-26
[GO:0044459] Plasma membrane part	1.09E-25
[GO:0005654] Nucleoplasm	1.73E-25
[GO:0005829] Cytosol	1.83E-23
[GO:0005887] Integral to plasma membrane	3.54E-21
[GO:0031226] Intrinsic to plasma membrane	6.36E-21
[GO:0043233] Organelle lumen	4.62E-20
[GO:0031974] Membrane-enclosed lumen	2.00E-18
[GO:0031981] Nuclear lumen	8.71E-18
[GO:0070013] Intracellular organelle lumen	1.06E-16

**Table 2:** Gene Ontology clustering of molecular functions

**Molecular function**	**False discovery rate**
[GO:0004672] Protein kinase activity	1.62E-14
[GO:0004713] Protein tyrosine kinase activity	3.31E-09
[GO:0008134] Transcription factor binding	4.72E-08
[GO:0046983] Protein dimerization activity	5.15E-08
[GO:0019899] Enzyme binding	6.45E-08
[GO:0019838] Growth factor binding	6.44E-07
[GO:0004714] Transmembrane receptor protein tyrosine kinase activity	7.72E-07
[GO:0042802] Identical protein binding	2.16E-06
[GO:0030528] Transcription regulator activity	2.95E-06
[GO:0019900] Kinase binding	4.94E-06

**Table 3:** Gene Ontology clustering of biological processes

**Biological process**	**False discovery rate**
[GO:0042127] Regulation of cell proliferation	5.99E-28
[GO:0010033] Response to organic substance	1.59E-24
[GO:0006796] Phosphate metabolic process	9.04E-22
[GO:0006793] Phosphorus metabolic process	9.04E-22
[GO:0043067] Regulation of programmed cell death	7.77E-21
[GO:0010941] Regulation of cell death	8.31E-21
[GO:0042981] Regulation of apoptosis	1.75E-20
[GO:0006468] Protein amino acid phosphorylation	3.14E-19
[GO:0010604] Positive regulation of macromolecular metabolic process	3.52E-19
[GO:0016310] Phosphorylation	1.02E-18

On the basis of the clustering results, when hepatoma cells occurred, the most significant changes were in cell membranes and cell nuclei. In addition, there were kinase and protein binding changes which were classic molecular functions of cell signaling transformation. All the changes caused by molecules were closely related to cancer, and the progress, proliferation and apoptosis of cells were all significantly clustered.

### Biopathways in hepatoma cells

When normal cells become cancerous, their expression profiles have a significant change, as do some genes. In this study, we selected differentially expressed genes to perform GO analysis of the KEGG PATHWAY with the aim of finding the changed pathways in hepatoma cells. Setting the false discovery rate at <0.05 and at least two genes in the signaling pathway as the limiting conditions, we obtained significantly changed pathways, which are shown in Table 4.

**Table 4:** **KEGG** bio**pathway changes in hepatoma cells**^**a**^

**Term**	**False discovery rate**
[hsa04010] MAPK signaling pathway	2.70E-09
[hsa05200] Pathways in cancer	9.90E-06
[hsa04510] Focal adhesion	0.001997
[hsa04660] T-cell receptor signaling pathway	0.002519
[hsa04640] Hematopoietic cell lineage	0.003705
[hsa05220] Chronic myeloid leukemia	0.020022
[hsa05212] Pancreatic cancer	0.034797
[hsa04350] TGF-β signaling pathway	0.041718
[hsa04722] Neurotrophin signaling pathway	0.046962

^a^KEGG, Kyoto Encyclopedia of Genes and Genomes; MAPK, mitogen-activated protein kinase; TGF-β, transforming growth factor β.

Compared with normal cells, the changes in hepatoma cells focus on signal transduction. These changes promote hepatoma cells resistant to the body’s own immune system and that interfere with the role of some drugs.

The focal adhesion pathway of hepatoma cells changes a lot. The focal adhesion pathway, which connects cells with the extracellular matrix, plays a key role in the motility, proliferation and differentiation of cells. Some of these connections serve as the connection structure between signaling receptors on the cell membrane and intracellular actin protein filaments, and even as direct signaling molecules, including various protein kinases and phosphatases. Therefore, changes in this pathway can block the normal signaling pathways in cells, so that the hepatoma cells changes sequentially.

Because of the blocking of signal transduction, a series of important cell signaling pathways change. The MAPK signaling pathway is an important intracellular signaling pathway regulating gene expression and plays an important role in the regulation of cell proliferation, differentiation and movement. The T-cell receptor signaling pathway is an important immune signaling pathway whose signals directly regulate T-cell proliferation. Therefore, the changes in this pathway may be the key for hepatoma cells to avoid autoimmunity. The changes in the TGF-β signaling pathway and the neurotrophin signaling pathway promote the formation of an independent group of hepatoma cells that can be distinguished from normal cells. It is worth mentioning that the hematopoietic cell lineage pathway also changes, which may make it easy to transfer the characteristics of the source. The final outcome of these changed signaling pathways changed the apoptosis pathway and the hematopoietic cell lineage pathway, so that the liver cells showed a unique pathology.

### Exploring the small effector molecules

cmap can be used to find the potential therapeutic drug candidates which are similar to the drug in hypoxic stimulus conditions and gene expression [15]. It is the first installment of a reference collection of gene expression profiles from cultured human cells treated with bioactive small molecules, together with pattern-matching software to mine these data [15,16]. To compare normal cells with hepatoma cells, the differentially expressed genes were divided into upregulation and downregulation. Compared with the differentially expressed genes in the cmap database by Gene Set Enrichment Analysis, we obtained some small molecules similar to normal cells or hepatoma cells. Twenty small molecules which had the strongest correlation with hepatoma cells (*P*-value minimum) were selected, and these are shown in Table 5 (all processing of small molecules and the effect of repression of low similarity are shown.

**Table 5:** **Small effector molecules**^**a**^

**cmap name**	**Enrichment**	***P***
Pyrvinium	−0.818	0.0001
Oxybuprocaine	−0.759	0.00692
Ticarcillin	−0.846	0.00735
Trifluridine	−0.696	0.01812
Molindone	−0.679	0.02335
Bambuterol	0.667	0.02751
Lovastatin	0.658	0.03141
Tiratricol	−0.645	0.03796
5255229	−0.848	0.0464
Thapsigargin	−0.65	0.08523
Dobutamine	−0.576	0.08934
α-Yohimbine	−0.629	0.10626
Orphenadrine	−0.456	0.11724
Amodiaquine	0.487	0.20486
Dorzolamide	0.477	0.2225
Fluorocurarine	0.474	0.22972
Anisomycin	−0.476	0.2304
SC-58125	−0.466	0.25202
W-13	0.642	0.25673
Levobunolol	−0.453	0.28421

^a^cmap, Connectivity Map database.

The results showed that the first small molecules could not simulate the state of normal cells well (enrichment <0.9). It is worth mentioning, however, that some small molecules returned to a state similar to that of normal cells with the use of drugs such as bambuterol (enrichment = 0.667) and lovastatin (enrichment = 0.658). In addition, we found some molecules with strong carcinogenic effects, such as pyrvinium (enrichment = −0.818) and ticarcillin (enrichment = −0.846).

## Discussions

HCC is a common and aggressive cancer that occurs mainly in men. The incidence is associated with gender, age and duration of the underlying liver disease. However, the most powerful risk factor is the existence of liver cirrhosis, regardless of its etiology [17]. High-volume alcohol intake is associated with the highest risk [18,19]. Aflatoxin intake also has a role in the genesis of HCC, but only in patients who have preexisting chronic hepatitis B [20]. Although great advancements have been made in the surgical treatment of HCC, tumor recurrence after surgery remains a key challenge for the clinical management of HCC patients [21].

In our study, we selected different individual tissues to analyze biochips with the aim of finding core HCC lesions (all data from Wang *et al*. [22]). Specifically, there were 621, 231, 29 and 37 reported probe sets representing 406, 153, 12 and 20 genes, respectively, from the studies of Lee *et al*. [23], Ye *et al*. [24], Iizuka *et al*. [25] and Kurokawa *et al*. [26], respectively. We excluded individual differences in order to find the common features, in which we found that as many as 9,775 genes that transcend individual differences affect the activity of the cells, showing that hepatoma cells indeed have some common features. Expression of the detoxification enzyme cytochrome P450 and enzymes involved in metabolism (AS3MT and HEXB) that are predominantly expressed in differentiated hepatocytes were downregulated in recurrent HCC samples. All tissue samples used in this study were approved and provided by the Tissue Repository of the National Cancer Centre, Singapore, and the study was conducted in accordance with the institution’s ethics committee policies.

The biopathways obtained after GO clustering of differentially expressed genes indicate that the commonality of hepatoma cells is tracked. Hepatoma cells infect intracellular and intercellular signal transduction through focal adhesion and cause abnormal expression of important intracellular signaling pathways (T-cell receptor signaling pathway, MAPK signaling pathway, TGF-β signaling pathway and neurotrophin signaling pathway). On the one hand, hepatoma cells block the body’s own immune response and affect cell apoptosis and proliferation. On the other hand, they change the morphological and behavioral characteristics of normal cells, transforming them into cancer cells and eventually leading to the occurrence of liver cancer. Hence, a better understanding of the clinicopathologic features and molecular aspects of HCC, as well as the ability to assess and stratify patients with different risk levels of disease recurrence at the time of diagnosis, would be extremely beneficial for the clinical management of HCC. This member gene set could serve as a pool of leading gene targets for the identification and development of novel diagnostic and therapeutic biomarkers to greatly improve the clinical management of HCC patients with different risks of recurrence after curative partial hepatectomy.

About 50 randomized controlled trials (RCTs) have been conducted to develop treatments for HCC patients, but transarterial embolization and tamoxifen administration are the only two options that have been best evaluated. The administration of tamoxifen, an estrogen receptor blocker, was initially reported to improve survival in patients with advanced HCC [27]. The activity of chemotherapy in patients with HCC is negligible. New agents with relevant activity are needed and will have to be tested within RCTs. On the basis of differentially expressed genes and information from the cmap database of small molecules, we found a series of small molecules. These small molecules can simulate to some extent the different states of hepatoma cells compared to normal cells, meaning that these small molecules may be able to repair disorders of liver metabolic pathways.

## Conclusions

The study has great significance for gene therapy and pharmacotherapy and provides a new treatment entry point and a potential new clinical drug for HCC patients.

## Competing interests

The authors declare that they have no competing interests.

## Authors’ contributions

DK, HC and WC carried out the molecular biology analysis, participated in the design of the study and clinical specimen collection, and drafted the manuscript. SL, HW, HL and QK carried out the clinical specimen collection, participated in the data analysis and performed the statistical analysis. ZL and XH conceived and designed the study, participated in data analysis and study coordination and helped to draft the manuscript. All authors read and approved the final manuscript.
